RETRACTED

# Pancancer Analysis of Neurovascular-Related NRP Family Genes as Potential Prognostic Biomarkers of Bladder Urothelial Carcinoma

**DOI:** 10.1155/2021/5546612

**Published:** 2021-04-15

**Authors:** Chao Deng, Hang Guo, Dongliang Yan, Tao Liang, Xuxiao Ye, Zuowei Li

**Affiliations:** Department of Urology, Shanghai Jiao Tong University Affiliated Sixth People's Hospital, Shanghai, China

## Abstract

**Background:**

Neurovascular-related genes have been implicated in the development of cancer. Studies have shown that a high expression of neuropilins (NRPs) promotes tumourigenesis and tumour malignancy.

**Method:**

A multidimensional bioinformatics analysis was performed to examine the relationship between NRP genes and prognostic and pathological features, tumour mutational burden (TMB), microsatellite instability (MSI), and immunological features based on public databases and find the potential prognostic value of NRPs in pancancer.

**Results:**

Survival analysis revealed that a low NRP1 expression in adrenocortical carcinoma (ACC), cervical squamous cell carcinoma and endocervical adenocarcinoma (CESC), low-grade glioma (LGG), and stomach adenocarcinoma (STAD) was associated with poor prognosis. A high NRP2 expression in bladder urothelial carcinoma (BLCA), kidney renal papillary cell carcinoma (KIRP), and mesothelioma (MESO) was associated with poor prognosis. Moreover, NRP1 and NRP2 were associated with TMB and MSI. Subsequent analyses showed that NRP1 and NRP2 were correlated with immune infiltration and immune checkpoints. Genome-wide association analysis revealed that the NRP1 expression was strongly associated with kidney renal clear cell carcinoma (KIRC), whereas the NRP2 expression was closely associated with BLCA. Ultimately, NRP2 was found to be involved in the development of BLCA.

**Conclusions:**

Neurovascular-related NRP family genes are significantly correlated with cancer prognosis, TME, and immune infiltration, particularly in BLCA.

## 1. Introduction

The growth and development of neovascular tissue or angiogenesis are critical for normal physiological processes. Therefore, dysregulation of the angiogenic process has been linked to tumour development and progression [1]. The vascular endothelial growth factor (VEGF) is a key factor involved in angiogenesis. VEGF messenger RNA (mRNA) is widely overexpressed in tissues and is associated with metastasis, recurrence, and prognosis [2]. In recent years, several drugs that inhibit the VEGF signaling pathway have been designed to treat cancer, including anti-VEGF monoclonal antibodies [3–6]. And neurovascular-related genes have been implicated in cancer development. There is a strong link between neural stem/progenitor cells (NSPCs) and endothelial cells (ECs) [7].

RETRACTED

Evidence suggests that neuropilins (NRPs), the VEGF receptors, are involved in tumourigenesis [8, 9]. NRPs participate in the development of the nervous system by functioning as receptors for axon guidance factors [10]. Several signaling pathways regulate neuronal development by targeting NRPs [11]. High expression of NRPs is closely associated with tumourigenesis and malignancy [12].

NRP1 and NRP2 are two isoforms of NRPs in mammals; studies have demonstrated their cancer-promoting potential [13]. For example, NRP2 is highly expressed in triple-negative breast cancers [14]. In prostate cancer, NRP2 expression is positively correlated with the Gleason grade [15]. In the bladder cancer, high expression of NRP2 is associated with chemoresistance and epithelial-to-mesenchymal transition and poor patient prognosis [16]. However, the expression and function of NRPs in different cancers are not fully known.

Herein, we comprehensively analysed the correlation of NRP expression with prognosis and tumour microenvironment landscape in 33 cancer types. Our findings reveal that NRPs may be a potential prognostic marker associated with immune infiltration, tumour mutations, and tumour microenvironment, particularly in bladder urothelial carcinoma (BLCA).

## 2. Materials and Methods

### 2.1. Analysis of Differential NRP1 and NRP2 Gene Expression in Human Cancer

RNA sequences, somatic mutations, and clinicopathological features of 33 cancers were downloaded from The Cancer Genome Atlas (TCGA) database. The data included 10,953 patients (10,967 samples). A pancancer analysis was performed on NRP1 and NRP2 mRNA expression levels in the Oncomine database (http://www.ONCOMINE.org). The threshold was set at *p* value < 0.05 and ∣fold change | >1.5. In addition, changes in NRP1 and NRP2 expression in different cancer types were determined using the R package “ggpubr” and the cBioPortal database (https://www.cbioportal.org). All data analyses were performed using version 4.0.3 of the R language package (https://www.r-project.org/).

### 2.2. Survival Analysis

The association of NRP1 and NRP2 with survival was assessed with the Kaplan-Meier method and log-rank test (*p* < 0.05). Patients were divided into high- and low-risk groups based on median expression levels of NRP1 and NRP2. Survival curves were created using “survminer” and “survivor” packages of R. Cox analysis was performed to explore the association of NRP1 and NRP2 with the prognosis of different cancers. A “forestplot” function was used to draw a forest plot whereas the “ggplot2” function was used to analyse clinicopathological features.

RETRACTED

### 2.3. Association of NRP Family Genes with Tumour Mutational Burden (TMB) and Microsatellite Instability (MSI) in Various Cancers

TMB was derived from a study published by Gentles et al. [17], and MSI was obtained from a study published by Bonneville et al. [18]. As in previous studies [19–21], statistical analyses were performed using the rank-sum test, and *p* values less than 0.05 were considered statistically significant; R software was used for plotting.

### 2.4. Association of NRP1 and NRP2 Expression with Immune Checkpoint-Related Genes in Different Cancers

As described in previous studies [22–27], the xCell method was used to perform immune score assessment. The immune checkpoint genes, *pDCD1*, *SIGLEC15*, *HAVCR2*, *IDO1*, *CD274*, *LAG3*, *CTLA4*, and *PDCD1LG2*, were analysed to examine the association of NRP1 and NRP2 with expression of immune checkpoint-related genes.

### 2.5. DNAss, RNAss, StromalScore, and ImmuneScore among Subgroups

The differentiated phenotype was rapidly lost during cancer progression, and progenitor and stem-cell-like characteristics were acquired [28]. RNAss based on mRNA expression and DNAss based on DNA methylation were utilized to measure the tumour stemness [29]. The ESTIMATE algorithm in the R language ESTIMATE package was used to estimate the ratio of immune to stromal components in the TME for each sample and is presented as two scores: ImmuneScore and StromalScore, which are positively correlated with immune and stromal components, respectively.

### 2.6. Integrative Data Visualization

The correlation of NRP1 and NRP2 with other genes was mapped using Cancer Regulome Tools (http://explorer.cancerregulome.org/). A *p* value > -log100 was considered statistically significant.

## 3. Results

### 3.1. NRP1 and NRP2 mRNA Levels in Pancancers

The flow chart of this study is shown in Figure 1. NRP1 and NRP2 were found to be widely expressed in human tissues (Figure 2(a)). The overall expression level of NRP1 did not significantly differ from that of NRP2 in human tissues (Figure 2(b)), suggesting good concordance between NRP1 and NRP2 expression in humans. Results of NRP1 and NRP2 mRNA levels in the Oncomine database are shown in Figures 2(c) and 2(d). We further assessed the expression of NRP1 and NRP2 in different cancers by analysing 730 normal samples and 10,327 fractional tumour samples in TCGA data sets (Figures 2(e) and 2(f)). Overall, whether NRP1 and NRP2 are highly or lowly expressed in tumour tissue was difficult to establish. The expression of NRP1 and NRP2 was different between normal tissue and tumour tissues in the brain and central nervous system cancers. Of note, the expression of NRP1 and NRP2 genes in some cancers was inconsistent in different databases. These inconsistencies may be caused by different gene extraction methods and biological mechanisms. These results demonstrate that NRP1 and NRP2 are differentially expressed in different tissues, suggesting they may have distinct roles in different tissues.

RETRACTED

### 3.2. Prognostic Value of NRP1 and NRP2 in Various Cancers

Next, we explored the prognostic value of NRP1 and NRP2 in various cancers in the TCGA database. We found that NRP1 and NRP2 expression was associated with the prognosis of various cancers. NRP1 was found to be a risk factor in different cancers, including ACC (HR 1.027, 95% CI 1.014-1.040, *p* < 0.001), CESC (HR 1.021, 95% CI 1.007-1.035, *p* < 0.003), GBM (HR 1.014, 95% CI 1.004-1.025, *p* = 0.009), LGG (HR 1.038, 95% CI 1.024-1.053, *p* < 0.0001), LIHC (HR 1.009, 95% CI 1.003-1.016, *p* = 0.0053), MESO (HR 1.011, 95% CI 1.003-1.020, *p* = 0.0062), and STAD (HR 1.018, 95% CI 1.010-1.026, *p* < 0.0001) (Figure 3(a)). In contrast, NRP1 was a protective factor in KIRC (HR 0.995, 95% CI 0.992-0.997, *p* < 0.0001). Further analysis showed that NRP2 was a risk factor in different cancers such as BLCA (HR 1.012, 95% CI 1.003-1.021, *p* = 0.0093), KICH (HR 1.178, 95% CI 1.008-1.375, *p* = 0.0390), KIRP (HR 1.048, 95% CI 1.015-1.081, *p* = 0.0040), LAML (HR 1.127, 95% CI 1.031-1.232, *p* = 0.0086), LGG (HR 1.012, 95% CI 1.002-1.021, *p* = 0.0168), LIHC (HR 1.015, 95% CI 1.001-1.029, *p* = 0.0400), MESO (HR 1.012, 95% CI 1.006-1.019, *p* = 0.0003), PAAD (HR 1.017, 95% CI 1.006-1.029, *p* = 0.0027), and STAD (HR 1.009, 95% CI 1.001-1.018, *p* = 0.0282) (Figure 3(b)). Survival analysis suggested that low NRP1 expression in adrenocortical carcinoma (ACC), cervical squamous cell carcinoma and endocervical adenocarcinoma (CESC), low-grade glioma (LGG), and stomach adenocarcinoma (STAD) was associated with poor patient prognosis. However, high NRP1 expression in kidney renal clear cell carcinoma (KIRC) predicted good prognosis (Figures 3(c)–3(g)). High NRP2 expression in BLCA, kidney renal papillary cell carcinoma (KIRP), and mesothelioma (MESO) was associated with poor prognosis (Figures 3(h)–3(j)).

### 3.3. Association of NRP1 and NRP2 Expression with TMB and MSI in Different Cancers

A high TMB influences immunotherapy sensitivity [28, 29]. Thus, we assessed the relationship between NPR2 expression levels and BLCA, kidney chromophobe (KICH), KIRP, acute myeloid leukemia (LAML), LGG, liver hepatocellular carcinoma (LIHC), MESO, pancreatic adenocarcinoma (PAAD), and STAD. This is because the expression of NRP1 and NRP2 correlated with the overall survival of such cancers (according to the results of one-way Cox and Kaplan-Meier survival analyses). The results showed that NRP1 expression was positively correlated with TMB in ACC and LGG but negatively correlated with the TMB of MESO, LIHC, and STAD expression (Figure 4(a)). NRP2 expression was positively correlated with the TMB of LAML and PAAD but negatively correlated with the TMB of MESO, KIRP, STAD, and LIHC (Figure 4(c)).

RETRACTED

In further analyses, it was found that NRP1 expression was significantly positively correlated with MSI in MESO but negatively correlated with MSI in STAD (Figure 4(b)). NRP2 expression was also significantly positively correlated with MSI in KIRC but negatively correlated with MSI in STAD (Figure 4(d)).

### 3.4. Coexpression of Immune Checkpoint Genes with NRP1 and NRP2 in Different Cancers

A coexpression analysis was performed to explore the correlation of NRP1 and NRP2 expression with immune checkpoint genes. In most cancers, NRP1 and NRP2 expression was found to be positively correlated with immune checkpoint genes (*CD274*, *CTLA4*, *HAVCR2*, *LAG3*, *PDCD1*, *PDCD1LG2*, *SIGLEC15*, and *TIGIT*) (Figures 5(a) and 5(b)). In BLCA, the NRP1 and NRP2 expression was negatively correlated with the *SIGLEC15* expression. In MESO, the *SIGLEC15* expression was negatively correlated with the NRP2 expression. In KIRC, *LAG3* and *PDCD1* expression levels were positively correlated with the NRP1 expression.

### 3.5. Association of NRP1 and NRP2 Expression with Immune Infiltration

Previously, we showed that low NRP1 expression in ACC, CESC, LGG, and STAD was associated with poor prognosis, whereas high NRP1 expression in KIRC predicted good prognosis. Moreover, high NRP2 expression in BLCA, KIRP, and MESO was associated with poor prognosis. Hence, the xCell approach was used to comprehensively assess the association of NRP family genes with immune infiltration (Figures 6(a) and 6(b)). We found that the NRP1 and NRP2 expression correlated significantly negatively with the T cell CD4+ Th1 expression in almost all of the cancer types. Infiltration of mast cells was positively correlated with the NRP1 expression in most of the cancer types. The high NRP1 expression in ACC, CESC, GBM, LGG, MESO, and STAD was associated with poor prognosis, suggesting that mast cell infiltration may be associated with NRP1 expression. In addition, high NRP1 expression was associated with higher stroma, microenvironment, and immune scores, as well as more endothelial cell infiltration in most tumours. A high NRP2 expression in BLCA and KIRP was associated with poor patient prognosis, while a high NRP2 expression in BLCA and KIRP implied depletion of T cell CD4+ central memory. Overall, these results suggest that the NRP1 and NRP2 expression is associated with alterations in immune gene expression and infiltration in different cancers.

RETRACTED

### 3.6. Association of NRP1 and NRP2 Expression with the TME in Various Cancers

The heterogeneity of TME across different cancers affects tumour drug resistance and modulates cancer progression and metastasis [30, 31]. Here, we further explored the association of NRP1 and NRP2 expression with the immune microenvironment of some cancers (LGG, BLCA, ACC, CESC, KIRC, KIRP, MESO, and STAD). The ESTIMATE algorithm was used to calculate, among other things, stem cell and immune cell indices in tumour cells. The expression of NRP family genes in BLCA and LGG was found to be correlated most significantly with RNAss, DNAss, StromalScore, ImmuneScore, and ESTIMATEScore (Figures 7(a) and 7(b)). Overall, the NRP1 and NRP2 expression was positively correlated with StromalScore, ImmuneScore, and ESTIMATEScore in most prognosis-related cancers (Figures 7(a)–7(h)). Conversely, the correlation of the NRP1 and NRP2 expression with RNAss and DNAss was heterogeneous across cancer types. In conclusion, expression of NRP family genes is associated with the TME of various cancers.

### 3.7. Association of NRP1 and NRP2 Expression with Clinicopathological Features in Various Cancers

Further analysis demonstrated that the NRP1 and NRP2 expression was correlated with clinicopathological features of several cancers (KIRC, LGG, STAD, BLCA, and KIRP) (Figures 8(a)–8(e)). In patients with KIRC and STAD, NRP1 expression was significantly correlated with ethnicity. The degree of NRP1 expression was higher in Blacks and Asians. In BLCA, NRP2 expression was higher in Asian populations compared to Caucasians. A high NRP1 and NRP2 expression was also found to be correlated with tumour diameter. In KIRC, a high NRP1 expression was associated with a larger tumour size, higher risk of distant metastases, and worse stage staging and grade staging. Similarly, a high NRP1 expression in STAD implied a worse grade staging. However, in LGG, a high NRP1 expression implied a better grade staging. Furthermore, in BLCA, NRP2 expression was associated with tumour size, stage staging, and worse grade staging. In KIPR, the NRP2 expression was higher in male patients.

### 3.8. Genome-Wide Association of NRP1 and NRP2 mRNA in Various Cancers

The previous results revealed that NRP1 might play important roles in KIRC and LGG, whereas NRP2 might play important roles in BLCA. Therefore, we analysed the association of KIRC, LGG, and BLCA with NRP1 and NRP2 in human genomic models (including gene expression, DNA methylation, somatic copy number, microRNA expression, somatic mutation, and protein level RPPA). The results showed that NRP1 was associated with genome-wide features in KIRC and LGG (Figures 9(a) and 9(b)), while NRP2 was broadly associated with genome-wide features in BLCA (Figure 9(c)).

RETRACTED

## 4. Discussion

Data obtained from pancancer analysis has the potential to guide tumour control strategies and design of therapies [32]. In recent years, genome-wide pancancer analysis has revealed mutations, RNA expression profiles, and immune profiles associated with tumour development. This has provided numerous biomarkers for the diagnosis and treatment of tumours [33].

In this study, we used different tools to analyse the expression of NRPs in different tumours and its association with mutations, TME, immune landscape, and prognosis. We found that neurovascular-associated NRPs can predict the prognosis of many cancers. Moreover, NRP1 and NRP2 were differentially expressed levels in different tissues. This suggests that they may play distinct roles in different cancers. Survival analysis demonstrated that a low NRP1 expression in ACC, CESC, LGG, and STAD was associated with poor patient prognosis, whereas a high NRP1 expression in KIRC predicted good prognosis. A high NRP2 expression in BLCA, KIRP, and MESO was associated with poor patient prognosis. Further analysis revealed that NRP1 and NRP2 were significantly associated with TMB and MSI in various cancers. Moreover, the NRP1 and NRP2 expression was positively correlated with the expression of immune checkpoint genes and immune infiltration. The expression level of NRPs was associated with the TME and clinicopathological features of cancers. Finally, genome-wide association analysis suggested that the NRP1 expression was closely associated with KIRC, whereas the NRP2 expression was closely associated with BLCA. Together with previous studies, we suggest that NRP2 may be involved in the development of various cancers, particularly BLCA.

NRPs are highly conserved, multifunctional transmembrane proteins that are unique to vertebrates and are involved in various physiological and pathological processes in the body [34, 35]. In mammals, there are two isoforms of NRPs (NRP1 and NRP2) that are functionally distinct and complementary. These genes are involved various biological processes such as neuroangiogenesis, cell migration, and immune regulation [36, 37].

A high NRP1 expression has been reported to be closely associated with tumourigenesis and progression, which is consistent with our findings [38, 39]. Using NRP1 antagonists, several studies have demonstrated the therapeutic potential of NRP1 in cancers [40]. Previous studies have also revealed that NRP1 modulates the function of various immune cells. In recent studies, NRP1 was found to regulate the stability and function of Tregs. It has also been reported to function as an antitumour immune inhibitor [41]. Anti-NRP1 treatment improved the efficacy of anti-PD-1 immunotherapy. This indicates that immunotherapy targeting NRP1 may have good clinical outcomes [42]. NRP1 has also been previously found to promote tumour angiogenesis, tumour proliferation, and migration [43–48]. Anti-NRP1 therapy can block tumour angiogenesis and upregulate the antitumour immune response [49–52]. Currently, anti-NRP1 therapy is used as a potential antitumour treatment option [42, 53]. In conclusion, the results of our study reveal that anti-NRP1 therapy has good clinical benefits.

RETRACTED

A high NRP2 expression in BLCA, KIRP, and MESO was associated with poor prognosis. Similar to our study, a high NRP2 expression in the bladder has been associated with chemoresistance and epithelial-to-mesenchymal transition [16]. In addition, a higher NRP2 expression has been reported in triple-negative breast cancers indicating that the NRP2 expression depends on the type of breast cancer [14]. Moreover, the NRP2 expression in prostate cancer is positively correlated with the Gleason grading [15]. NRP2 is closely related to the immune system [12]. The xCell algorithm was to first provide indirect data on the expression pattern of NRP2 in B cells, NPRs, natural killer cells, and T cells. Recent studies have shown that NRP2 regulates various processes such as cell migration and antigen migration in the immune system [12]. Similarly, this study reveals that NRP2 influences immune processes. NRP2 has also been found to be closely associated with metastasis and BRAFV600E in thyroid cancer [54]. Downregulation of NRP2 has been shown to influence epithelial-mesenchymal transition by affecting phosphorylation signaling pathways [54]. This suggests a potential association of NRP2 expression with the TME and gene mutations.

Energy metabolism is interconnected, coupled to insulin signaling, and linked to the release of metabolic hormones from adipose tissue. Understanding the diverse roles of energy metabolism should prevent and treat various human diseases such as diabetes, obesity, and cancer [55]. Previous studies have found that NRP1/2 may be involved in energy metabolism [56, 57]. Diabetes is an energy metabolism-related disease that can lead to multiple systemic pathologies [58–61]. And diabetes is closely associated with neurovascular disease [62–65]. Therefore, we propose the bold hypothesis that NRP1/2 may also influence tumour prognosis through energy metabolism-related pathways.

RETRACTED

However, there are limitations to this study that warrant further exploration. Firstly, the present study does not demonstrate how NRPs influence tumour growth and developmental processes by affecting the immune microenvironment or the TME, as well as other pathways. Secondly, *in vivo* and *in vitro* experiments should be performed to substantiate our results and clarify the impact of NRP expression on tumourigenesis development. Further studies at cellular and molecular levels would be beneficial to elucidate the specific functional mechanisms of NRPs in different cancer types. Thirdly, future well-designed studies are needed such as single-cell RNA sequencing. Further improvements in precision would be beneficial to prevent systematic bias at the cellular level. Therefore, future cohort studies and population-based case-control studies are necessary to examine the mechanisms involved.

## 5. Conclusion

In conclusion, neurovascular-related NRP family genes are significantly correlated with the prognosis, TME, and immune profiles of tumours, especially in BLCA. Therefore, NRPs may be used as a marker for predicting the prognosis of various tumours. Besides, NRPs hold great promise as a potential target for tumour therapy.

## Figures and Tables

**Figure 1:** Flow chart for this study.

**Figure 2:** NRP1 and NRP2 mRNA levels in pancancers. (a) NRP1 and NRP2 expression levels in human tissues. Darker colours indicate higher levels of expression. (b) Overall expression of NRP1 and NRP2 in human tissues. (c) Differential in NRP1 expression in cancer and normal tissues in the Oncomine database. The number in each small rectangle represents the number of high or low expression of NRP genes in each cancer. Red (high expression) and blue (low expression) shading indicates the proportion in each cancer tissue. (d) Box plots from TCGA's database demonstrating differential expression of NRP1 expression in different tumour and normal samples. (e) Differential expression of NRP2 expression in cancer and normal tissues in the Oncomine database. (f) Box plots from TCGA's database demonstrating differential expression of NRP2 expression in different tumour and normal samples.

**Figure 3:** Prognostic value of NRP1 and NRP2 in pancancers (a, b). Association of NRP1 and NRP2 with the prognosis of different tumours in the univariate Cox analysis. (c–j) Association of NRP1 and NRP2 expression with the prognosis of different tumours as determined from Kaplan-Meier survival curves.

**Figure 4:** Correlation analysis between NRP1 and NRP2 gene expression and TMB and MSI in pancaner: (a) correlation between NRP1 and TMB; (b) correlation between NRP1 and MSI; (c) correlation between NRP2 and TMB; (d) correlation between NRP2 and MSI.

RETRACTED

**Figure 5:** Coexpression of immune checkpoint genes with NRP1 (a) and NRP2 (b) in pancancers. Heat map of immune checkpoint-related gene expression in different tumour tissues, where the horizontal axis represents different tumour tissues and the vertical axis represents immune checkpoint-related gene expression.

**Figure 6:** Heat map of Spearman correlation analysis between the xCell/EPIC immune score and the NRP family gene expression in multiple tumour tissues, where the horizontal axis represents different tumour tissues, the vertical axis represents different immune scores, different colours represent correlation coefficients, negative values represent negative correlation, and positive values represent positive correlation (^∗^*p* < 0.05, ^∗∗^*p* < 0.01, ^∗∗∗^*p* < 0.001). Significance of the two sample groups by Wilcoxon test.

**Figure 7:** (a–h) Correlation analysis of NRP1 and NRP2 expression with tumour microenvironment in pancancer (LGG (a), BLCA (b), ACC (c), CESC (d), KIRC (e), KIRP (f), MESO (g), and STAD (h)).

**Figure 8:** Correlation analysis of NRP1 and NRP2 expression with clinicopathological features in pancancer. The distribution of clinical characteristics in different groups of samples, where the horizontal axis represents the different groups of samples and the vertical axis represents the percentage of clinical information contained in the sample of the corresponding group. Significant differences were analysed by the chi-square test, where the magnitude of the value was taken as -log10 (*p* value); ∗ means that there is a significant difference in the distribution of the clinical characteristic in the corresponding two groups (*p* < 0.05).

**Figure 9:** Genome-wide association of NRP1 and NRP2 mRNA in pancancer (Regulome program). NRP1 is broadly associated with genome-wide features in KIRC (a) and LGG (b). NRP2 is also found to be broadly associated with genome-wide features in BLCA (c).

## Data Availability

All data was obtained from the public database described in Materials and Methods.

## Abbreviations

ACC: Adrenocortical carcinoma
BLCA: Bladder urothelial carcinoma
BRCA: Breast invasive carcinoma
CESC: Cervical squamous cell carcinoma
CHOL: Cholangiocarcinoma
COAD: Colon adenocarcinoma
DLBC: Lymphoid neoplasm diffuse large B-cell lymphoma
ESCA: Esophageal carcinoma
GBM: Glioblastoma multiforme
LGG: Brain lower grade glioma
HNSC: Head and neck squamous cell carcinoma
KICH: Kidney chromophobe
KIRC: Kidney renal clear cell carcinoma
KIRP: Kidney renal papillary cell carcinoma
LAML: Acute myeloid leukemia
LIHC: Liver hepatocellular carcinoma
LUAD: Lung adenocarcinoma
LUSC: Lung squamous cell carcinoma
MESO: Mesothelioma
OV: Ovarian serous cystadenocarcinoma
PAAD: Pancreatic adenocarcinoma
PCPG: Pheochromocytoma and paraganglioma
PRAD: Prostate adenocarcinoma
READ: Rectum adenocarcinoma
SARC: Sarcoma
SKCM: Skin cutaneous melanoma
STAD: Stomach adenocarcinoma
TGCT: Testicular germ cell tumours
THCA: Thyroid carcinoma
THYM: Thymoma
UCEC: Uterine corpus endometrial carcinoma
UCS: Uterine carcinosarcoma
UVM: Uveal melanoma.
